# Innovative Application of Artificial Intelligence in the Field of Innovation and Entrepreneurship of College Students in Internet Colleges and Universities

This article has been retracted.

**DOI:** 10.1155/2022/3538755

**Published:** 2022-08-08

**Authors:** Liping Bai, Fei Sun, Wenhao Wang

**Affiliations:** ^1^Graduate School, Lyceum of the Philippines University, Manila 1002, Philippines; ^2^Innovation and Entrepreneurship School, Hangzhou Vocational and Technical College, Hangzhou 31000, Zhejiang, China; ^3^Graduate School, The University of Manila, Manila 1002, Philippines

## Abstract

With the promotion and development of artificial intelligence, the computer major has become a hot major in innovation and entrepreneurship education. It is increasingly essential to carry out a refined evaluation of creativity and venture education to achieve professional differentiation. The purpose of this paper is to study and explore the innovative use of AI in the field of innovation and entrepreneurship of college students in Internet universities. In the article, AI is first introduced. AI is inherently a novel instrument of human praxis, a tool of productivity that embodies human ability and volition. Then we analyze the innovation and venture education on the ground of the BP neural network, and finally, we conduct an empirical study on the innovation and venture on the ground of the BP neural network. Innovation and entrepreneurship refer to entrepreneurial activities based on one or several innovations in technological innovation, product innovation, brand innovation, service innovation, business model innovation, management innovation, organizational innovation, market innovation, and channel innovation. The report analyzes the influencing factors of creative venture education and designs an evaluation model of creative venture education. The test shows that the output of the BP neural network is the actual value, the real worth is reasonable, and the desired worth is also reasonable. The maximum error between the two is 1.64%. The results tend to be generally satisfactory. The BP neural network model can highly generalize students' creative venture abilities, increasing the practical application value and research scope of BP neural networks.

## 1. Introduction

In the context of informatization and globalization, multifield integration is the development trend of innovation and entrepreneurship education. Creative and entrepreneurial education is an educational concept and mode of simultaneous cultivation and development of thinking and ability, practice, and theory. Creative and entrepreneurship education refers to the educational content related to future development. In order to cultivate creative and enterprising personnel, innovation and venture education are closely integrated with talents. Innovative and entrepreneurial higher education is widely concerned by countries all over the world and has profoundly influenced the research and growth of tertiary education. Especially, the cultivation of innovative and pioneering education for students in different professional fields has not yet formed an interactive model and evaluation system of innovative and pioneering education in line with national conditions. Therefore, it is in line with the need for educational reform to study the assessment mechanism of creative and entrepreneurship education in computer science.

It expands the evaluation theory of creative venture education and provides new thoughts for the evaluation of creative venture education for computer science students, which is beneficial to the construction and growth of the subject. The article proposes an improvement policy for innovation and entrepreneurship education in computer science, which enriches the theory of innovation and venture education in colleges and universities and the theory of employment guidance for college students, and broadens the theory of advanced education. At the same time, a set of assessment indicators system for creative venture education of computer science majors is proposed, which provides a new direction of thinking and research ideas for the subsequent related evaluation research. Based on the perspective of the BP neural network, this paper analyzes the data of graduates majoring in computer science. It provides advice on innovation and entrepreneurship education for computer science students. It has important practical significance for the development of innovation and entrepreneurship education in colleges of computer and software. This facilitates the development of computer science students' job creation and self-improvement needs.

The innovation of this paper is as follows: (1) it introduces artificial intelligence that is a new technical science that studies and develops simulation methods, techniques, and application systems, (2) it analyzes the innovation and entrepreneurship education based on BP neural network, and (3) it conducts experimental research on innovation and entrepreneurship based on the BP neural network. This paper discusses the influencing factors of innovation and entrepreneurship education and constructs an evaluation model for innovation and entrepreneurship education.

## 2. Related Work

According to the research progress in foreign countries, different researchers have conducted corresponding cooperative research in innovation and entrepreneurship. GerardoBarroso-Tanoira and Tanoira [1] came up with a plan. They promoted students' creativity, innovation, and entrepreneurial motivation. They were based on interventions in business companies to improve the performance of employees by using critical and inventive thought [1]. Promoting social innovation and entrepreneurship is a panacea in the long run. This will fuel the country's development agenda and address the country's social problems. Thus, Kumar et al. [2] explored the prospects for social innovation and entrepreneurship in the country. They took a practice-based approach with reference to contemporary social issues [2]. The essence of technological innovation and the birth of great digital technology, digital information platform, and digital information technology infrastructure have greatly influenced the spirit of innovation and entrepreneurship culture. Nambisan et al. [3] aimed to appreciate the need for research on the digital transition of the economy to include multiple and interlevel analyses, including thoughts and perceptions from multiple fields/disciplines, and to explicitly acknowledge the role of digital technologies in transforming tissue and society relations [3]. However, these scholars lack a certain technical analysis of innovation and entrepreneurship research. Therefore, artificial intelligence technology needs to be introduced to analyze innovation and entrepreneurship.

Some scholars also have some research results in artificial intelligence technology. Lu et al. [4] planned to produce an intelligence learned tool named brain intelligence (BI) model. The model generates fresh thoughts about incidents without experiencing them by the use of imaginative artificial beings [4]. Hassabis et al. [5] examined the historical exchange between the fields of artificial intelligence and animal neuroscience research and highlights current developments in artificial intelligence technology. This progress has also been influenced by neurocomputing studies in humans and other animals [5]. Li et al. [6] highlighted the opportunities and challenges of leveraging AI for smart 5G networks. They also envisioned AI-enabled 5G cellular networks that will make the acclaimed ICT enabler a reality [6]. However, these scholars did not research and discuss the innovative application of artificial intelligence in the field of innovation and entrepreneurship of college students in Internet colleges and universities but only discussed its significance unilaterally.

## 3. Innovative Application Methods of Artificial Intelligence in the Field of Innovation and Entrepreneurship of College Students in Internet Colleges and Universities

Innovative entrepreneurship education refuses to depart from traditional expertise but emphasizes innovative expertise, which is the basis and rationale for creative discipline [7]. Artificial intelligence technology is a new tool.

It not only liberates human physical strength but also releases human brain power. Professional education is also inseparable from innovative training, so innovative training is the sublimation and expansion of traditional professional knowledge [8]. The main research direction of artificial intelligence is to use intelligent machines to enhance the power and effectiveness of human beings in various tasks of changing nature and governing society. The key features of creative entrepreneurial education compared to traditional education are as follows [9]. First, creative entrepreneurial education has the connecting function of bonding [10]. In the 1990s, creative and enterprising higher education in China received widespread attention. The basic condition for a breakthrough in the development of tertiary education in China is innovative and entrepreneurial higher education. Higher education is constantly receiving new ideas and nutrients, while innovation and entrepreneurship education is constantly innovating and developing. The two are closely linked and have important implications for education. Second, innovation and entrepreneurship education conforms to social and economic development and needs. It is very important to establish a new outlook on career choices. The employment problem of college students today is quite serious. Innovation and entrepreneurship teaching under the guidance of professional education has adapted to the requirements of the current social development trend. The innovative spirit and entrepreneurial ability have a huge impact on the students and have far-reaching significance. It is essential to replace students' thoughts and consciousness of passive acceptance and to cultivate their learning habits of independent entrepreneurship and development. In the format of imitation, competition and planning are more approachable. Among them, creative entrepreneurial education in the form of business practice meets the fundamental needs of creative entrepreneurial education. However, the research on creative applications in the domain of creative venture for college students in Internet universities still needs to be analyzed. Therefore, this paper analyzes and researches the creative venture of college students according to the BP neural network algorithm in artificial intelligence algorithm.

### 3.1. Artificial Intelligence

AI is inherently a novel vehicle for human praxis. The vehicle of productivity embodies human ability and volition. For instance, facial identification is already widely used as a tool in airports, scenic spots, train stations, and so on as shown in Figure 1. In such places where there is a high flow of people, intelligent recognition machines “scan faces” to increase the speed of passenger flow and reduce congestion. Some ticket inspectors at the windows are also relieved from mechanical labor.

AI was a consequence of the physicalization of human intellect. Another major avenue of technology evolution is the study of mimicking another animate entity [11], as shown in Figure 2. In the long evolution of tools, humans first realized the evolution of tools by simulating other organisms. After the simulation of other creatures reaches a certain level, they gradually seek to simulate themselves, from easy to difficult, from simple to complex, and gradually realize the evolution and upgrading of tools [12]. The artificial intelligence produced by the materialization of thinking and thinking results is the product of the long-term development of nature and the practice of human society.

### 3.2. Innovation and Entrepreneurship Education Based on BP Neural Network

#### 3.2.1. BP Neural Network Model

An artificial neural network does not need to determine the mathematical equation of the mapping relationship between input and output in advance. As an intelligent information processing system, the core of an artificial neural network to realize its function is an algorithm. BP neural network is a multilayer feedforward network trained by error backpropagation (referred to as error backpropagation). Its basic idea is gradient descent. It uses the gradient search technique in order to minimize the error mean square error between the actual output value of the network and the expected output value.

The BP neural network cleverly applies this machine learning algorithm, which is more suitable for various network technologies. Error backpropagation calculations are also introduced [13]. According to the properties and regularities of the function, the neural network can automatically learn past experiences from the provided complex data samples. The BP algorithm is a unique and attractive program, and the neural network is a challenging technological frontier technology, so the two are combined into a BP neural network [14]. The neural network has the characteristics of high self-adaptation, self-organization, and self-learning. According to the laws and characteristics of functions, the neural network conducts scientific and reasonable analysis of complex problems and finds the most effective strategies and methods to solve them [15] as shown in Figure 3.

#### 3.2.2. BP Neural Network Structure

The BP network is to add several layers (one or more layers) of neurons between the input layer and the output layer. These neurons are called hidden units. They have no direct connection with the outside world. But changes in its state can affect the relationship between input and output. Each layer can have several nodes. The input layer belongs to the front-end part, and the hidden layer belongs to the middle part. The output layer belongs to the end part, and they together form the BP neural network. The input vector is the beginning of data import and occupies an important position; then the formula *a*=(*a*_1_, *a*_2_,…*a*_*m*_,…*a*_*p*_)^*D*^ is expressed; and assumption (*a*_0_=−1) can be added at the same time. The hidden layer belongs to the middle part, which directly affects the training changes in the neural network. The output vector is the result of data export, which has great significance. The expression formula is *b*=(*b*_1_, *b*_2_,…*b*_*m*_,…*b*_*q*_)^*D*^, and hypothesis (*b*_0_=−1) can be added. The introduction of the threshold through the output layer neurons is of critical significance and has a huge impact on the terminal part.

The output layer output vector is *u*=(*u*_1_, *u*_2_,…*u*_*h*_,…*u*_*k*_)^*D*^. The weight matrix between the input layer and the hidden layer is because the input layer is an important beginning of receiving data, and the hidden layer is an important process of transmission and change. The weight matrix generated between the two has a great effect on the BP neural network. The matrix expression is *l*=(*l*_1_, *l*_2_,…*l*_*h*_,…*l*_*q*_)^*D*^. And because the output layer is the export port of the data, the generation between it and the hidden layer is of great significance to the BP neural network, so the matrix expression is *e*=(*e*_1_, *e*_2_,…*e*_*n*_,…*e*_*k*_)^*D*^.  Figure 4 shows the principle flow of the BP neural network.

Inside the network, the mathematical relationship between each part plays a huge role. The first is the front-end part, also called the input layer, which passes and acts on the front-end part [16].

(1) $$\begin{array}{c} u_{h}=g\left({\text{net}}_{h}\right),\;h=1,2,\ldots ,p,\\ {\text{net}}_{h}=\sum_{n=0}^{q}e_{nh}b_{n},\;h=1,2,\ldots ,p. \end{array}$$

The second is the middle part, also known as the hidden layer, which affects the middle part through *b*_*n*_ and net_*n*_.

(2) $$\begin{array}{c} b_{n}=g\left({\text{net}}_{n}\right),\;h=1,2,\ldots ,q,\\ {\text{net}}_{n}=\sum_{m=0}^{q}nl_{mn}a_{m},\;n=1,2,\ldots ,q. \end{array}$$

The unipolar sigmoid function is a class of functions, and the transfer function *g*(*a*) is applied to the inner part of the neural network. Both *g*(*a*) can choose the unipolar sigmoid function [17].

(3) $$\begin{array}{c} g\left(a\right)=\frac{1}{1+e^{-a}}. \end{array}$$

Continuous functions generally have continuity and derivability, which makes the function application range wider. Then *g*(*a*) has this property [18].

(4) $$\begin{array}{c} g{}^{\prime }\left(a\right)=g\left(a\right)\left[1-g\left(a\right)\right]. \end{array}$$

Another category of functions is the bipolar sigmoid function. Functions also have their own characteristics and have a wide range of applications [19].

(5) $$\begin{array}{c} g\left(a\right)=\frac{1-e^{-a}}{1+e^{-a}}. \end{array}$$

The final three-layer BP neural network is composed of the above parts.

The calculation process of the BP neural network consists of a forward calculation process and a reverse calculation process. The input mode is processed layer by layer from the input layer through the hidden unit layer and turned to the output layer. The state of neurons in each layer only affects the state of neurons in the next layer. If the desired output cannot be obtained at the output layer, it turns to backpropagation. It minimizes the error signal by modifying the weights of each neuron.

The BP training algorithm is the process of introducing the algorithm and training on the basis of the BP neural network. The important steps are as follows:

 Step 1: The first step is to set variables and parameters. *a*_*h*_=[*a*_*h*1_, *a*_*h*2_,…, *a*_*hq*_],  (*h*=1,2,3,…*p*) are input vectors, and *p* is the total number of samples [20].

(6) $$\begin{array}{c} E_{QM}\left(p\right)=\left[\begin{array}{cccc} E_{11}\left(p\right) & E_{12}\left(p\right) & \cdots & E_{1M}\left(p\right)\\ E_{21}\left(p\right) & E_{22}\left(p\right) & \cdots & E_{2M}\left(p\right)\\ \vdots & \vdots & \vdots & \vdots \\ E_{Q1}\left(p\right) & E_{Q2}\left(p\right) & \cdots & E_{QM}\left(p\right) \end{array}\right]. \end{array}$$

The above expression is the weight vector between the beginning part and the middle part *M* during the *p*-th iteration.

(7) $$\begin{array}{c} E_{MN}\left(p\right)=\left[\begin{array}{cccc} E_{11}\left(p\right) & E_{12}\left(p\right) & \cdots & E_{1N}\left(p\right)\\ E_{21}\left(p\right) & E_{22}\left(p\right) & \cdots & E_{2N}\left(p\right)\\ \vdots & \vdots & \vdots & \vdots \\ E_{M1}\left(p\right) & E_{M2}\left(p\right) & \cdots & E_{MN}\left(p\right) \end{array}\right]. \end{array}$$

Formula (7) is the weight vector between the middle part *M* and the middle part *N* at the *p*-th iteration.

(8) $$\begin{array}{c} E_{NO}\left(p\right)=\left[\begin{array}{cccc} E_{11}\left(p\right) & E_{12}\left(p\right) & \cdots & E_{1O}\left(p\right)\\ E_{21}\left(p\right) & E_{22}\left(p\right) & \cdots & E_{2O}\left(p\right)\\ \vdots & \vdots & \vdots & \vdots \\ E_{N1}\left(p\right) & E_{N2}\left(p\right) & \cdots & E_{NO}\left(p\right) \end{array}\right]. \end{array}$$

After the loop iteration of *p* produces the output result, the actual output value is

(9) $$\begin{array}{c} b_{h}\left(p\right)=\left[b_{h1}\left(p\right),b_{h2}\left(p\right),\ldots ,b_{hp}\left(p\right)\right],\;\left(h=1,2,3\ldots p\right). \end{array}$$

The expected output value is *t*_*h*_=[*t*_*h*1_, *t*_*h*2_,…, *t*_*h*3_],  (*h*=1,2,3 … *p*).

Step 2: During the network initialization process, *E*_*QM*_(*p*), *E*_*MN*_(*p*), and *E*_*NO*_(*p*) are each assigned a nonzero random number, and *p* = 0.
Step 3: It inputs the data of sample *a*_*h*_ because the sample data is the basic data of neural network training, which is closely related to the network, and set *p* = 0 at the same time [21, 22].
Step 4: The association between the weights of the middle part and the end part and the output vector is
  (10) $$\begin{array}{c} l_{o}\left(po\right)=b_{ho}\left(p\right)\;o=1,2,3,\ldots ,o. \end{array}$$
Step 5: It calculates the error *W*(*p*) based on *t*_*h*_ and *b*_*h*_(*p*). Assuming that the set requirement error is met, it jumps to the eighth step 8. Assuming that the set requirement error is not met, it jumps to step 6.
Step 6: The number of parameter iterations is calculated inside the BP neural network, and then *p* + 1 is compared with it [23, 24]. Assuming that the former is greater than the latter, it adjusts to step 8. Assuming the latter is greater than the former, it requires computing neuron local gradients.
  (11) $$\begin{array}{c} \varphi_{o}^{o}\left(p\right)=b_{o}\left(p\right)\left(1-b_{o}\left(p\right)\right)\left(t_{o}\left(p\right)-b_{o}\left(p\right)\right). \end{array}$$
Step 7: Inside the BP neural network, the weights between the front part, the middle part, and the end part have a huge influence [25, 26].
  (12) $$\begin{array}{c} \Delta E_{no}\left(P\right)=\beta \varphi_{o}^{o}\left(p\right)l_{n}^{N}\left(p\right)\;n=1,2,3\ldots N,\\ E_{no}\left(p+1\right)=E_{no}\left(P\right)+\Delta E_{no}\left(P\right)\;o=1,2,3,\ldots o,\\ \Delta E_{mn}\left(P\right)=\beta \varphi_{n}^{N}\left(p\right)l_{m}^{M}\left(P\right)\;m=1,2,3\ldots M,\\ E_{mn}\left(p+1\right)=E_{mn}\left(P\right)+\Delta E_{mn}\left(P\right)\;n=1,2,3\ldots N. \end{array}$$
Step 8: Neural network training samples take time. Assuming it is completed, it exits the training process directly; if not, it adjusts to step 3.

#### 3.2.3. Improvement of BP Neural Network

BP neural networks offer benefits, but they also have the following disadvantages:

1. There is a contradiction between the local minimum and the global optimum, and it is difficult to obtain the global optimum
2. If the neural network is trained more often, the drawbacks are a slow conversion rate and low productivity
3. Only on the basis of theoretical guidance can the scientific and accurate prediction results of the neural network be guaranteed, especially the determination of the number of hidden layer nodes that requires theoretical guidance [27, 28]
4. There is a contradiction between learning new samples and forgetting old samples, while neural networks tend to forget old samples

To address the shortcomings of neural networks, algorithms need to be tweaked and modified [29, 30].

The momentum term needs to be added. The learning rate of *β* is closely related to the BP neural network algorithm. If the value of *β* is too large, the network will converge faster, but it will cause instability. A value of *β* is too small to avoid instability, but the convergence is too slow. So it introduces the momentum term, among which *γ*  is the momentum term.

(13) $$\begin{array}{c} \Delta E_{mn}\left(P\right)=\gamma \Delta E_{mn}\left(p-1\right)+\beta \varphi_{n}\left(P\right)l_{n}\left(P\right). \end{array}$$

Considering formula (13) as a time series with *d* as a variable, *d* is from 0 to *p*; then

(14) $$\begin{array}{c} \Delta E_{mn}\left(P\right)=\gamma \sum_{d=0}^{p}s^{p-d}\varphi_{n}\left(d\right)l_{n}\left(d\right). \end{array}$$

The learning rate needs to be adjusted. It sets the learning rate to *β*, and the overall error decreases after changing the weights. *β*=*τβ* (*τ* < 0) can be changed through the learning rate, and the weights also change to varying degrees. This leads to a downward adjustment in the total error, thus illustrating the role of the adjustment of the learning rate.

It selects the odd function as the excitation function. The odd function is a kind of function and has its own uniqueness. The BP neural network operation can be accelerated by taking an odd function as the excitation function. Hyperbolic tangent functions are a common odd function.

(15) $$\begin{array}{c} g\left(V\right)=a\;\tanh\left(bv\right)\\ =s\left[\frac{1-\exp\left(-bv\right)}{1+\exp\left(-bv\right)}\right]\\ =\frac{2s}{1+\exp\left(-bv\right)}-s. \end{array}$$

In the practical application of the artificial neural network, most of the neural network models use the BP network and its variations. It is also the core part of the forward network, which embodies the essence of an artificial neural network. The BP network is mainly used in the following four aspects. (1) function approximation: it trains a network to approximate a function with input vectors and corresponding output vectors; (2) pattern recognition: it uses a pending output vector to relate it to the input vector; (3) classification: it classifies the appropriate way defined by the input vector; and (4) data compression: it reduces the dimension of the output vector for easy transmission or storage.

This paper takes computer science students as the object of study. On the basis of sorting out the relevant literature at home and abroad, it firstly focuses on the assessment indicator system of creative entrepreneurial education for computer science students, then carries out the actual analysis of creative entrepreneurial education assessment according to BP neural network model, and finally expects to provide theoretical support and countermeasure suggestions for creative entrepreneurial education for computer science students. The technical route of the research is shown in Figure 5.

## 4. Experimental Results of Innovative Application of Artificial Intelligence in the Field of Innovation and Entrepreneurship of College Students in Internet Colleges and Universities

An artificial neural network is a nonlinear system that models complex problems involving multiple factors. The artificial neural network does not need to establish a mathematical model, and it uses the weights and thresholds of neurons in each layer to represent the training data to obtain experience. The model can summarize implicit rules from a large number of complex data samples with unknown patterns through continuous learning and training and then obtain evaluation results, which is superior to traditional evaluation methods. If it evaluates the same type of problem, it only needs to input sample data into the model and get the result. In the evaluation process, it avoids human subjective intervention, and the evaluation results are more accurate. In addition, it uses the MATLAB professional platform to make the evaluation model of innovation and entrepreneurship education for computer majors more scientific and accurate.

### 4.1. Influencing Factors of Innovation and Entrepreneurship Education

This paper mainly takes the undergraduate graduates majoring in computer science from a university as the research object. It is dominated by the distribution of questionnaires on the “Questionnaire Star” online platform, supplemented by mail and paper questionnaires. A total of 1,902 questionnaires were collected. After screening, a total of 1,768 valid questionnaires were obtained, accounting for 92.9%. Among the graduates in this survey, there are 1,198 males, accounting for 67.76%, and 570 females, accounting for 32.24%. The sample distribution is shown in Table 1.

It implements the basic principles of comprehensiveness, science, comparability, representativity, and operability. At the same time, it fully considers the characteristics of the school, the family education background of the students, and the campus innovation and entrepreneurship environment and other influences on the school's teaching system to set indicators. This paper mainly explains the main content of innovation and entrepreneurship education evaluation from four aspects: school background, students' comprehensive ability of professional knowledge, students' comprehensive ability of practical operation, and students' comprehensive ability of development. It is shown in Figure 6.

At the same time, this paper also uses Cronbach's coefficient test method. The homogeneity test is a standard test, which is authoritative in the industry. On this basis, the content consistency of the questionnaire survey was studied. It also assumes that the higher the confidence value of the questionnaire on the survey, the more stable the measurement results. The reliability value accepted by experts is 0.7. According to the conclusions of the reliability analysis, as shown in Table 2, the reliability values of all survey questions are over 0.7, and the consistency of the questions is high. And there is considerable credibility, indicating that the problem is set reasonably and meets the relevant requirements.

### 4.2. Basic Ideas of Innovation and Entrepreneurship Education Evaluation

The basic idea of applying the BP neural network to the evaluation of innovation and entrepreneurship education for computer majors: First, it determines the input vector and output vector and takes the evaluation index data as the input vector. It then uses the scoring value obtained by the Delphi method as the output vector data. Second, it designs the BP neural network structure, which covers the selection of initial values, the number of network layers, and so on. Then, it uses the collected specific data to complete the establishment, training, and detection of the BP neural network to achieve the prediction function. It compares the actual output obtained with the predicted result. If the deviation range is exceeded, it can continue to dynamically adjust the weights and thresholds of the network until the specified deviation requirements are met. Finally, the trained BP neural network is used as a practical evaluation tool, and the BP neural network model becomes an evaluation model for computer science students' creative venture education.

### 4.3. Model Design of Innovation and Entrepreneurship Education Evaluation

#### 4.3.1. Determining the Number of Neural Network Layers

It passes through a process of infinitely pinching the BP network of the hidden layer, and the final result realizes the mapping from *n* dimension to *m* dimension. Kolmogorov's theorem reveals that even a three-layer neural network has a wide range of applications and high performance. Thus, a three-layer nerve neck network can also approach the ensemble feature with any accuracy as long as the amount of implicit level nodes is not limited. Increasing the number of hidden layers has advantages and disadvantages. So, to get low training error, the best choice is to create a three-layer neural network model.

#### 4.3.2. Determining the Number of Neurons in Each Layer

It determines the number of neurons in the input layer. The number of neurons in the input layer is an important feature inside the neural network, and on this basis, the two are equivalent and unified. The evaluation index is 21, which are the actual length of time engaged in social development, family members with entrepreneurship-related background, joining innovation or entrepreneurship associations, innovation experience, high school entrance examination results, test scores for the development of innovation ability, declaration of invention patents, declaration of software copyrights, core talents in software product development, a noncore talent in software development, participating in school-level competitions (“Internet +,” Create Youth, Challenge Cup) and winning awards, participating in provincial college students' innovative development plans, participating in national competitions and win awards, participating in provincial competitions and winning awards, compiling business plans and research reports, participating in centralized technology innovation training camps sponsored by venture funds, participating in corporate R&D plans, actively writing scientific research journal papers, and actively carrying out innovation and entrepreneurship online courses to obtain computer technology and software professional and technical qualification examination certificates. So the number of neurons in the input layer is *n* = 21.

It determines the total number of neurons in the hidden layer and the output layer. The actual output value of the network is unique, so the total amount of the output layer neurons is also unique, that is, *m* = 1. By comparing the total amount of neurons in the concealed layer with the total amount of neurons in the import and export layers, it is vulnerable to interference and conflicts from the external environment. If the number is smaller, there is also less information. If the number is large, it will lead to poor fault tolerance. The training time is too long, and there is “overfitting.”

Through the analysis of Figure 7, the number of neurons in the hidden layer is 4, 5, 6, 7, 8, 9, 10, 11, 12, and 13, and it is found that the training error decreases continuously at this time, and there is a connection. When the test error is 10, 11, and 12, the fluctuation first rises and then falls. Overall analysis, when the number of hidden layer neurons is 11 is the best choice.

#### 4.3.3. Determining the Learning Rate

The learning rate directly affects the efficiency of the training and testing of neural networks. When the learning rate is large, the weights are large, and the convergence is fast, resulting in large network fluctuations. A small learning rate leads to uncertain network efficiency and slow convergence.

The evaluation results analyze the error and training times of Figure 8 and finds that the learning rate is 0.01.

#### 4.3.4. Determining the Training Function

Six representative training functions are Levenberg–Marquardt, Rprop, ScaledConjugate-Gradient, OnestepSecant-Algorithm, gradient drop, and gradient drop with the self-adaptive rate of learning and impulse factor. The training results of different training functions are compared with respect to the total number of training steps and performance, and the performance advantages of different training functions are highlighted as shown in Table 3.

#### 4.3.5. Data Initialization

According to the evaluation index system of innovation and entrepreneurship education for computer majors, the BP neural network that has been trained, verified, and tested has become an effective prediction model. According to the Delphi method, the corresponding student categories with corresponding innovation and entrepreneurship ability scores are summarized, as shown in Table 4.

### 4.4. Implementation of BP Neural Network

It first takes 1,768 computer science students' innovation and entrepreneurship evaluation data as the input vector of the BP neural network model. It takes the corresponding scores of the innovation and entrepreneurship ability of computer majors as the output vector and imports them into the neural network model to train the model. Then it verifies the accuracy of the model and finally tests and evaluates the model.

The parameters and training results of the BP neural network model show that the training process and verification process of the BP neural network and the overall test effect are ideal. The *R*-value is equal to 0.95359 in the training process fitting regression, 0.91759 in the validation process fitting regression, and 0.94128 in the overall process fitting regression. The fitting effect of the BP neural network model is ideal, indicating that the experimental data and the model have certain discipline and rationality. The neural network fitting regression comparison analysis chart also further verified the accuracy of the experiment.

According to the analysis in Figures 9 and 10, after the training of the improved BP neural network is completed, some test data are randomly chosen to test the BP neural neck module to get the corresponding evaluated values of creative entrepreneurial training in computer science. The overall comparison of the real versus expected values of the network output is analyzed, and it is clear that the actual values are basically the same as the expected values, without substantial changes. This also shows the reliability of the neural network model and the reasonableness of the collected data. The real and expected values of the trained neural network are basically the same. Only in the 9th, 10th, 15th, 16th, 19th, and 20th ordinal numbers, there are local fluctuations, which are also within the admissible limits.

## 5. Discussion

The comparative analysis leads to the desired result of comparing the real versus desired results. Students with higher evaluation scores have a solid foundation in computer science. Computer majors should take solid professional knowledge and participate in national competitions and college student training programs as the leading role in carrying out innovation and entrepreneurship education. In the computer major, the outstanding performance of the students' professional ability is to obtain the advanced qualification certificate in the software level examination. At the same time, according to the data collected by the author, the proportion of students who obtained the advanced qualification certificate in the computer technology and software professional and technical qualification examination is quite small, which shows that the advanced qualification certificate of the software proficiency examination has a heavyweight. From the analysis of the data collected by the school, the professional knowledge of the computer majors of the school is relatively solid.

## 6. Conclusions

BP neural network can effectively evaluate students' creative and entrepreneurial skills. In this paper, we first designed the structure of BP neural network, then completed the establishment, practiced and tested of the BP neural network, and finally determined the innovative entrepreneurial education evaluation model. This BP neural network module effectively evaluates the creative and entrepreneurial skills of students and broadens the application value and research field of the BP neural network. This article has actively explored the creative entrepreneurial education assessment of computer specialty. Further improvement and research are still needed in the future, and theoretical research should be strengthened. There is still room for further improvement of the evaluation model of innovation and venture education constructed in this article. It also fully combs domestic and foreign research literature to pave the way for comprehensive research in this field. It comprehensively selects research data and can carry out different levels of innovation and entrepreneurship education evaluation research.

## Figures and Tables

**Figure 1:** Artificial intelligence applications.

**Figure 2:** Intelligent materialization of artificial intelligence.

**Figure 3:** Topological structure diagram of BP neural network model.

**Figure 4:** Principle of BP neural network.

**Figure 5:** Technology roadmap.

**Figure 6:** Main content of innovation and entrepreneurship education evaluation.

**Figure 7:** The relationship between the number of neurons in the hidden layer and the error.

**Figure 8:** Comparison of results of different learning rates.

**Figure 9:** Actual and expected values of the neural network after training 1.

**Figure 10:** The actual and expected values of the neural network after training 2.

**Table 1:** Distribution of sample structure of graduate questionnaires.

Gender	Number of samples	Percentage (%)
Male	1,198	67.76
Female	570	32.24
Total number	1,902	100

**Table 2:** Reliability analysis of questionnaires.

Attributes	Coefficient value
Student background	0.851
Students' professional ability	0.729
Students' practical ability	0.779
Students' ability to develop	0.702

**Table 3:** Comparison of training results of different training functions.

Algorithm	Training steps	Properties
Levenberg–Marquardt	987	4.79
Rprop	46	2.41
ScaledConjugate-Gradient	987	1.79
OnestepSecant-Algorithm	987	1.61
Gradient descent method	987	2.31
Gradient descent with adaptive learning rate and momentum factor	181	2.61

**Table 4:** Division of innovation and entrepreneurship ability and student category.

Student category	Specific instructions	Ability corresponding value
Entrepreneur	—	100
Postgraduate student	Admitted to “985 Project” universities or study abroad	
Researcher	Guaranteed to “985 Project” colleges and universities	

Postgraduate student	Admission to “211 Project” universities or “Double First-Class” universities	90–99.9
Researcher	Guaranteed to “211 Project” universities or “Double First-Class” universities	
Employed person	Monthly salary of more than 10,000 yuan	

Postgraduate student	Admitted to general colleges	80–89.9
Researcher	Guaranteed to ordinary colleges and universities	
Employed person	Monthly salary 5,000–10,000 yuan	

Employed person	Monthly salary 3,000–4,999 yuan	70–79.9

Unemployed	—	<70

## Data Availability

Data sharing is not applicable to this article as no new data were created or analyzed in this study.
